The article "Dental Age Estimation Using Multiphoton Microscopy: A Potential Tool for Forensic Science" was published in 2022. Journal: Biomed Res Int.

# Dental Age Estimation Using Multiphoton Microscopy: A Potential Tool for Forensic Science

**DOI:** 10.1155/2022/3328818

**Published:** 2022-07-29

**Authors:** Juan M. Bueno, Rosa M. Martínez-Ojeda, Ana C. Fernández-Escudero, Francisco J. Ávila, Manuel López-Nicolás, María D. Pérez-Cárceles

**Affiliations:** ^1^Laboratorio de Óptica, Instituto Universitario de Investigación en Óptica y Nanofísica, Universidad de Murcia, Campus de Espinardo (Ed. 34), Murcia, Spain; ^2^Departamento de Medicina Legal y Forense, IMIB-Arrixaca, Facultad de Medicina, Universidad de Murcia, Murcia, Spain; ^3^Departamento de Física Aplicada, Universidad de Zaragoza, Zaragoza, Spain; ^4^Departamento de Dermatología, Estomatología, Radiología y Medicina Física, Universidad de Murcia, Murcia, Spain

## Abstract

Normal aging affects the different structures of teeth, in particular, the dentine. These changes are useful in forensic disciplines as a tool for age estimation. Although multiphoton (MP) microscopy has been used to explore dental pieces, a relationship between age and MP response of the human dentine has not been proposed yet. The relationship between MP signals and natural dentine aging is investigated herein. An index of age (INAG) combining two-photon excitation fluorescence (TPEF) and second harmonic generation (SHG) images has been used to quantify these changes. The results show that the INAG significantly decreases with age. Moreover, peritubular dentine size and collagen internal properties are also modified with age. This information confirms the usefulness of this technique in forensic age estimation after disasters (natural or manmade) with a lack of comprehensive fingerprint database. Courts and other government authorities might also benefit from this tool when the official age of individuals under special circumstances is required for legal or medical reasons.

## 1. Introduction

Age estimation is important in forensic sciences and essential in crime scenes or mass disasters involving unknown human bodies, as well as in asylum-seeking or unaccompanied minors in the absence of proper documents [1, 2]. This is also relevant for the investigator to limit the search for individuals within a missing person list and to minimize efforts during judicial or legal proceedings. Although anthropological analyses based on skeletal remains are useful tools, age estimation is a complex and challenging task [1, 3]. Among others, individual variations in biological maturity, metabolic changes, rates of pathologic conditions, and environmental factors have variable influence on the aging process [3].

Among the different procedures used in forensic age estimation, the use of teeth has been reported to be useful [4]. Dental pieces survive inhumation well, endure high temperatures and humidity, and show less variability than skeletal age [1]. In addition, dentition development is better than other available aging indicators. Different tools have been reported to estimate age in teeth, including morphological, biochemical, and spectroscopic analyses, among others [4–10].

The article "Dental Age Estimation Using Multiphoton Microscopy: A Potential Tool for Forensic Science" was published in 2022. Journal: Biomed Res Int.

Enamel, dentine, and pulp are the three major components of the human tooth [11]. The former is the hard outer surface that serves as protection and is made of mineralized calcium salts. This is separated from the dentine by the dentine-enamel junction. Dentine is the bulk of the tooth tissue, with porous appearance, that helps to protect the innermost pulp [12]. It is a mineralized tissue mostly composed of tubules (~0.8-2.5 *μ*m in diameter) which are responsible for hydration and tooth sensory responses, among others. These dentinal tubules are covered by collagen type I fibrils [13]. Nerves, blood vessels, and odontoblasts are within the dental pulp chamber. The latter are cells that originate the collagen-based mineralized tissue that forms the dentine. This is known as dentinogenesis, a process that occurs throughout life [12].

Since nonlinear optical responses of dental tissues were investigated in the 90's [14–16], different studies have used multiphoton (MP) microscopy to extract information on dental structures using three noninvasive imaging modalities: Two-photon excitation fluorescence (TPEF), second harmonic generation (SHG), and third harmonic generation (THG) [17–19]. Both TPEF and SHG microscopy are based on the quasisimultaneous absorption by the sample of pairs of infrared photons and the emission of visible photons with less (TPEF) or equal (SHG) energy of the sum of the two incident photons. Compared to regular microscopy, these techniques provide high resolution images, larger penetration depth within the tissue, inherent confocality, and reduced photodamage [17, 18]. In addition, regular staining procedures used to facilitate the visualization of features are not required when using MP imaging. Biological structures containing collagen, elastin, and myosin are efficient MP emitters. Then, the particular composition and structure of both enamel and dentine are especially suited for being analyzed with this technique.

Kao reported that dentine exhibited TPEF, SHG, and THG signals. However, in enamel only, TPEF and THG signals were detected [20]. These results were later corroborated by Chen and collaborators [21]. Three-dimensional morphological details of the dentinal tubules were analyzed by combining SHG and THG signals [22], and the prism structure of enamel was successfully revealed through THG images [23]. Structural details of the dentin-enamel junction have been also explored using MP imaging [21, 24]. This transitional zone presented an irregular line with absence of signal. Moreover, the intensity of the dentine SHG images was found to decrease from the inner dentinal areas to the junction. A multimodal microscope combining MP and coherent antistokes Raman scattering (CARS) imaging has also been proposed [25, 26]. In areas nearby the dentine-enamel junction, CARS images were much sharper than TPEF ones and showed a better sectioning performance. The combination of both techniques has recently been reported to provide useful information on the chemical composition in healthy and demineralized enamel [27]. Abnormalities and dental diseases have also been explored with MP microscopy [23, 28, 29]. These included spot lesions, cracks, and caries stages.

The article "Dental Age Estimation Using Multiphoton Microscopy: A Potential Tool for Forensic Science" was published in 2022. Journal: Biomed Res Int.

On the other hand, SHG signals from collagen-based tissues are sensitive to the polarization state of the incident light [30, 31]. Although some imaging procedures have been combined with polarization to evaluate dental pieces and demonstrate clinical feasibility [32–34], the potential of polarization-resolved SHG microscopy to explore optical anisotropy and internal organization of dental structures is scarce in literature [35].

Despite the amount of procedures used to estimate tooth age [4–10, 36], most of them have used electronic microscopy, and results therein do not always agree to each other. In addition, although a number of studies on dental pieces have used MP microscopy, analyses on aging using this imaging technique have not been found by these authors.

Dentine suffers a variety of changes with age [11, 36, 37] that might be tracked and objectively classified by means of MP imaging microscopy. In particular, dentinal tubules are surrounded by a mineralized peritubular zone (peritubular dentine), embedded in an (intertubular) organic matrix [11, 12]. As dentine ages, different structural changes are produced, including an increase in the mineral content, the secondary dentine formation, and the obturation of the tubules by peritubular dentine, what result in a decrease in sensation to pain, cold, and hot. A detailed description of age-related alterations of dentine can be found in [38] and references therein.

Therefore, it is crucial to improve the existing procedures by incorporating alternative tools to conduct more reliable age assessment methods for the various global populations. In that sense, the aim of this work is to explore the relationship between MP signals (TPEF and SHG) and aging in the human dentine. Structural arrangements, as well as changes in the internal organization of the dentinal tubules, are also analyzed. Results here obtained might be of interest in forensic age estimation.

The article "Dental Age Estimation Using Multiphoton Microscopy: A Potential Tool for Forensic Science" was published in 2022. Journal: Biomed Res Int.

## 2. Methods

### 2.1. Multiphoton Microscope and Experimental Procedure

A custom polarization-resolved MP microscope was used for the purpose of the present work [39]. A schematic of the instrument is depicted in Figure 1. A mode-locked Ti/Sapphire laser (Mira900f, Coherent) was used as excitation source (wavelength (*λ*) = 800 nm). The laser repetition rate was 76 MHz, and the output pulse width was ~150 fs. A polarization state generator (PSG) placed in the illumination pathway was used to modulate the incident polarization state as explained below. The XY galvanometer mirrors (VM1000, GSI) scanned the beam across the sample. The backscattered emitted MP signal from the specimen was collected via the same objective used for illumination (Nikon ELWD ×20, numerical aperture (NA) = 0.5) and detected by a photomultiplier tube (PMT, R7205-01, Hamamatsu). A long-pass (FGL435, Thorlabs Inc.) or a narrow-band spectral filter (FB400-10, Thorlabs Inc.) allowed for the isolation of TPEF and SHG signals, respectively. A step-by-step *Z*-motor (PI C-136) coupled to the microscope objective controlled the locations of interest within the sample.

The PSG is composed of a fixed horizontal linear polarizer (P_H_), a rotatory half-wave plate (*λ*/2). This configuration was designed to generate sets of linear polarization states. Further details on this can be found in [31, 39].

Image acquisition (at 1 Hz frame rate) and postprocessing were carried out using custom-written codes in LabVIEW™ and MATLAB™, respectively. The image size for all images was 180 × 180 *μ*m^2^. The averaged laser power at the sample was always the same along the entire experiment (40 mW). This was controlled through a neutral density filter (NDF). The present experiment was divided into two parts as described in the next sections.

### 2.2. Samples

Human dental samples (*N* = 9) were provided by the Clínica Odontológica de la Universidad de Murcia (Hospital Universitario Morales Meseguer, Murcia, Spain). Teeth were normal (i.e., free of any dental pathology) and extracted due to orthodontic reasons. Only the age (from 19 to 82 years old) and the sex of the patients were known, and the rest of details remained unknown in order to protect patients' confidentiality. Of the dental pieces analyzed, 4 corresponded to men and 9 to women. The mean ages of the former and the latter were 44.8 ± 21.6 and 47.4 ± 23.5 (years ± standard deviation), respectively. There was no statistically significant differences between age according to sex (*p* = 0.867, Mann–Whitney *U* test). The protocol was approved by the Ethical Research Committee of Murcia University (ID-2035/2018).

The article "Dental Age Estimation Using Multiphoton Microscopy: A Potential Tool for Forensic Science" was published in 2022. Journal: Biomed Res Int.

Each tooth was sectioned into two parts along the buccolingual and longitudinal axis with a diamond saw and immediately stored in 0.9% phosphate-buffered saline (PBS) solution. For MP imaging, specimens were placed in a bottom-glass dish filled with saline solution with the internal open section in an upside-down position lying in contact with the cover-glass. The specimens were not labeled with exogenous markers, what is intended to preserve their integrity.

### 2.3. Fiber Size and External Organization

For this part of the experiment, the PSG was set to generate horizontally polarized light. MP images from the dentine were acquired. Imaged zones were randomly chosen across coronal dentinal areas located close to the pulp. This avoids any possible influence of the dentinal location on the size of the peritubular dentine. In particular, for each dental piece, five pairs of TPEF and SHG images were recorded.

The peritubule size was computed from SHG images as follows. For every image, the greyscale was thresholded for a better visualization of the features; so, we can detect the orientation of the elongated tubules by computing the Hough transform [40]. Then, with this information, different cross-sections perpendicular to those structures were made for each image. These sections presented maximum and minimum intensity values corresponding to the tops and the valleys of the tubular areas, respectively. The size of these peritubules was calculated as the distance between consecutive valleys and expressed in microns (*μ*m).

In addition, the external organization of the peritubular dentine was also studied. For this, the structure tensor was used. Details on this can be found in [41]. In brief, this is an objective method to analyze the spatial organization of tissues composed of fiber-like structures. This mathematical tool provides numerical parameters for both the level of organization (known as structural dispersion, SD) and the preferential orientation of the fibers (if this exists). In particular, if the fibers are quasialigned along a particular direction, SD ≤ 20°. For a nonorganized distribution, SD > 40°. Values in between are associated to a partially organized arrangement.

Moreover, the parameter used in this work to quantify the structural information as a function of age was the contrast of the MP signals. This has been named as Index of aging (INAG) and is defined as [42]

(1) $$\begin{array}{c} \text{INAG}=\frac{{\tilde{I}}_{\text{SHG}}-{\tilde{I}}_{\text{TPEF}}}{{\tilde{I}}_{\text{SHG}}+{\tilde{I}}_{\text{TPEF}}}. \end{array}$$

The article "Dental Age Estimation Using Multiphoton Microscopy: A Potential Tool for Forensic Science" was published in 2022. Journal: Biomed Res Int.

### 2.4. Polarimetric Assessment and Internal Organization

For the second part of the experiment, the PSG was used to generate the different polarization states required to compute the value of the ratio of hyperpolarizabilities, *ρ* [43, 44], whereas SD informs on the organization of the collagen at an external scale (i.e., microscale) and is quantified through the structure tensor, and this parameter *ρ* is related to the internal structure (i.e., nanoscale) [30, 45]. In particular, as previously reported by Ávila et al. [44], three polarimetric SHG images are required to experimentally compute *ρ*: two of them to get the magnitude and the third one to provide the sign. The former is related to the internal order (the higher the value the higher the organization) and the latter to the intrinsic chirality of the collagen [46, 47]. In this work, the linear polarization states used to acquire SHG images were horizontal, vertical, and linear at 60° [44].

For a better understanding, Figure 2 presents an illustrative example of the entire experimental procedure used in this work.

## 3. Results

### 3.1. Dentine External Organization

Figure 3 shows representative SHG images of the dentine-enamel junction and the dentine of one of the dental pieces used in the present experiment. This signal is a result of the collagen component of the dentine [21]. The irregular interface between dentine and enamel is clearly visualized due to the nonappearance of SHG signal at the enamel (probably due to the absence of noncentrosymmetric proteins) [24]. Moreover, in both images, the structure of the dentinal peritubules is visible. These tubules are perpendicular to the inner boundary of the enamel layer (Figure 3(a)).

Changes in the size of the peritubular structure with age can qualitatively be seen in Figure 4. This presents SHG images corresponding to the dentine of two different dental pieces aged 19 and 82. For each specimen, the size was computed as described above. The averaged values are depicted in Figure 5. There was a significant linear increase of this parameter as a function of age (*R* (Pearson′s correlation) = 0.86, *p* = 0.003).

On the other hand, it is readily visible that the peritubular dentine presents a fairly well aligned distribution (see Figures 3 and 4). In order to check if the variation in width with age leads to a change in dentinal external organization, the SD has been computed using the structure tensor as described in Methods. This parameter informs about the degree of organization of a tissue composed of elongated structures (such as the dentine). The values of SD for all the samples involved in the experiment are shown in Figure 6. It can be observed that SD is always, close to, or below 20°, what is associated with a highly-organized structure [41]. This behavior indicates that despite peritubular dentine grows in size with age, the quasiparallel external arrangement is maintained.

The article "Dental Age Estimation Using Multiphoton Microscopy: A Potential Tool for Forensic Science" was published in 2022. Journal: Biomed Res Int.

### 3.2. Nonlinear Signals in Dentine

Figure 7 depicts TPEF and SHG images of the dentine for a dental piece. For a direct comparison, the images shared the same color scale. Despite both MP signals are produced, a direct observation reveals differences in the intensity within each pair of images: SHG signal was much lower than that corresponding to TPEF. In particular, for this specimen the ratio SHG/TPEF averaged across the image was 0.57 ± 0.02. For the set of samples here involved, the values ranged between a maximum of 0.62 and a minimum of 0.39. Dentinal peritubules, although present in both images, are better outlined in the TPEF image.

The relationship between SHG and TPEF signal might be associated to changes in the dentine with age. To explore these changes, the INAG was computed for each pair of SHG/TPEF images. As an example, Figure 8 depicts the spatially resolved INAG maps for two dental pieces with different age (24 and 60). A simple visualization shows that the map for the younger specimen presents a lighter color (orangish).

INAG values as a function of age for all samples involved in the present experiment are depicted in Figure 9. Each symbol represents the value averaged across all five imaged areas for the corresponding specimen. From this plot, it can be observed that all samples present negative INAG values (below -0.27). In addition, these experimental data also show a statistically significant linear relationship (*R* = 0.83, *p* = 0.006) with age. The slope of the linear regression with age is -0.003 units/year. Statistical differences between men and women were not found for this set of samples.

### 3.3. Dentine Internal Collagen Organization

Figure 10 presents two sets of polarimetric SHG images corresponding to samples aged 19 and 60 (each image was recorded for a different incident polarization state, as indicated in Methods). For direct visual comparisons, the images within a row share the same color code. For each set of images, the corresponding maps of the parameter of internal organization (i.e., *ρ*) were computed pixels-by-pixel (both magnitude and sign).  Figure 11 shows these maps for the samples of the previous figure. The averaged *ρ* values across the images were −1.25 ± 0.20 and −2.69 ± 0.50, as indicated in the insets.

The parameter *ρ* was then computed for all samples involved in the experiment.  Figure 12 shows the results. Values reduce with increasing age, and they are in range between -1.05 and -2.96. Moreover, a significant linear correlation between *ρ* and age was found (*R* = 0.95 and *p* < 0.0001): *ρ* = –0.02,·age–1.03. Unlike external arrangement structure that seems to be maintained (see Figure 6), internal organization increases (i.e., becomes more negative) with increasing age.

The article "Dental Age Estimation Using Multiphoton Microscopy: A Potential Tool for Forensic Science" was published in 2022. Journal: Biomed Res Int.

## 4. Discussion

The analysis of dental structures is a fundamental tool in forensic sciences [4, 8, 9]. In particular, dental age estimates is of great importance under certain circumstances where individuals cannot be identified visually or by other regular means. Although different procedures have been reported to determine tooth age [5–10], most of them do not provide enough accuracy. As an alternative method, here, we demonstrate MP imaging microscopy as a valuable tool to conduct further investigations on age estimation in human dentine.

In the process of getting old, changes take place in the tooth. However, although many of them are normal age-related changes, others are associated with disease and trauma [11, 36, 37]. In particular, tubular dentine structure is greatly affected [38]. Experiments using the ac-impedance technique found differences which were attributed to peritubular deposition on the inner walls of dentinal tubules [7]. The permeability of coronal dentine was much lower in the teeth of old patients than that in young teeth [48]. An increase in human teeth fragility with age and suggested changes in the dentine collagen has been reported [49]. Very recent experiments have also shown a relationship between a number of trace elements and the age of the teeth [50].

In spite of these changes, the principal cause for the age-related degradation in dentinal properties seems to be still unclear [11], and further exploration of the mechanisms of aging is needed. In that sense, this work goes a step forward in that direction, and age-related changes in the dentine have been analyzed using MP microscopy. In our experiment, pairs of TPEF-SHG images were successfully acquired from dentinal areas as a function of age. Although dentine was shown to emit both types of MP signals, the signal from TPEF images was higher than that from SHG images.

To the best of our knowledge, SHG signals (no images) from human dentine were early detected by Altshuler et al. [14]. Since demineralization did not modify SHG efficiency, this signal was attributed to the presence of collagen within the dentine. In 2000, Kao and coworkers reported SHG images from dentine for the first time [51]. Initial low quality images were later improved to show the tubular structure [20]. Some years later, TPEF and SHG images from dentine were presented by Cheng and coauthors [21]. Our findings agree well with those previous experiments. However, a relationship between dentine MP signals and aging is lacking in literature.

The article "Dental Age Estimation Using Multiphoton Microscopy: A Potential Tool for Forensic Science" was published in 2022. Journal: Biomed Res Int.

Herein, we have proposed an index (named as INAG) to explore whether MP signals correlate with age in the human dentine. Results reveal that INAG values are always negative, and there exists a linear decrease of this parameter with age (Figure 9, slope: -0.003 units/year). On average, by age 80, the index INAG will be 58% larger than that corresponding to a person aged 20. Negative values indicate that for each analyzed dentine area, SHG intensity is always lower that the corresponding to TPEF signal. Moreover, according to the INAG definition, an elder person would have a more negative index since the dentine of such an individual is expected to have lower collagen content.

The combination of TPEF-SHG image pairs has also been useful for different applications in the past. It was used to quantify collagen destruction within the corneal stroma during infectious processes [52] and to objectively assess skin aging changes (i.e., photoaging), both ex-vivo [42] and in-vivo [53]. Our results are coherent with the latter in the sense that INAG is able to objectively detect changes in the human dentine as a function of age.

It is interesting to notice that despite the passing years, the degree of external organization (i.e., SD) of the dentinal tubules is fairly maintained with age as a well-organized arrangement (Figure 6). On the opposite, a significant increase in tubular size with age was found, with an increase rate of 0.03 *μ*m/year (Figure 5).

The dentinal tubule density and diameter have been explored by different authors as a function of different factors (location, age, depth, primary/permanent teeth, tooth type,…) using scanning electron microscopy [5, 54, 55]. However, values are variable, and they do not always agree to each other.

In 1994, Koutsi et al. reported that the dentinal tubular diameter in primary molars from children ranged from 0.96 *μ*m at the superficial dentine to 1.29 *μ*m at deeper zones [56]. Variations with depth were also found later; although, the values were larger: between 2.4 *μ*m and 4.28 *μ*m [55]. However, no differences between primary second molars (from children aged 9 to 12 years) and permanent third molars (from individuals aged 18 to 23 years) were found. This diameter in primary molars was lower than that of permanent teeth. For children aged 9-11 years old, the average diameter was different when comparing first (0.794 *μ*m) and second molars (1.0 *μ*m) [57]. For 4-14 year-old children, Sikanta and coauthors reported a size of 1.44 *μ*m in molars and 1.15 *μ*m in incisors [58].

The article "Dental Age Estimation Using Multiphoton Microscopy: A Potential Tool for Forensic Science" was published in 2022. Journal: Biomed Res Int.

It must be taken into account that the tubules of this previous literature were imaged in the transversal direction (i.e., across the direction perpendicular to the tubules), and they have been reported to decrease in size with age. This experimental condition clearly differs from ours, since MP images are acquired along a longitudinal direction (i.e., along the axes of the tubules). It also is important to remind that SHG imaging does not visualize the tubules themselves, but the peritubular collagen covering those tubules. Then, the increase in peritubular width (as tubules reduce) reported herein seems to be coherent with those findings. This width ranged on average 4.30 *μ*m in young teeth, to 6.02 *μ*m in dental pieces aged 75-82 years.

For the size of the set of teeth here used, we did not found differences in sex. However, this study will be extended in the next future to a much larger set of samples in order to explore the possible relationship between normal tooth aging and sex. Moreover, an in-depth analysis of pathological samples will be also of great interest.

On the other hand, polarimetric SHG images show that the dentine of older teeth is more sensitive to polarization. This can be qualitatively observed by comparing the differences in SHG intensity in the images of Figure 10. This higher sensitivity to polarization with increasing age is quantitatively shown through the parameter *ρ* in Figures 11 and 12. This parameter significantly decreases with age (-0.02 units/year). This indicates that the collagen-based structure of the dentine does not present the typical age-related structural modifications that usually include collagen denaturation processes and loss of organization [30, 59–61]. Instead, normal aging leads to an increase in the internal collagen organization (or alternatively, high/*ρ*/[i.e., absolute value of *ρ*]) [47]. Although further analyses involving additional SHG polarimetric methods and samples of wider age groups are required, this increase in/*ρ*/might be closely associated to internal (i.e., molecular) collagen properties such as circular dichroism, chirality, and orientations of the longitudinal axis of the triple helix [46, 62].

To conclude, we applied MP microscopy (both TPEF and SHG images) to visualize changes in the human dentine as a function of age. We demonstrated that the index INAG can be used to quantify age-related changes. Significant changes in the diameter of the peritubular dentine were also found. In addition, polarimetric SHG microscopy has shown an increase in polarization sensitivity with age and a significant relationship with the ratio *ρ*. Our results suggest that MP imaging can be used as an accurate and effective quantitative tool for age determination. Forensic sciences would especially benefit from this method, since dental age estimation becomes of importance in cases involving people without any identity, bone remains, and paleontological studies.

The article "Dental Age Estimation Using Multiphoton Microscopy: A Potential Tool for Forensic Science" was published in 2022. Journal: Biomed Res Int.

## Figures and Tables

**Figure 1:** Schematic of the polarimetric MP microscope used for the purpose of this work, see details in the text. NDF: neutral density filter; PSG: polarization state generator; DIC: dichroic mirror; PMT: photo multiplier tube.

**Figure 2:** Example of the experimental procedure in one of the samples involved in the present study.

**Figure 3:** SHG microscopy images showing representative areas of the enamel-dentine junction (a) and the dentine (b).

**Figure 4:** SHG microscopy images of the dentine of two teeth of different age (19 (a) and 82 (b) years old). Differences in the size of the peritubules can easily be observed.

**Figure 5:** Relationship between age and peritubular width. Each symbol corresponds to the mean value for the corresponding specimens across all imaged dentinal areas. Error bars indicate the standard deviation. Black line represents the best linear fit to the data (size = 0.03^∗^age + 3.47).

**Figure 6:** Structural dispersion of the peritubular dentine as a function of age. Each symbol represents the value averaged across all SHG images within a sample. Error bars correspond to the standard deviation.

**Figure 7:** SHG (a) and TPEF (b) microscopy images of the dentine of a dental pieces aged 19. Blue and green pseudocolors were used to denote SHG and TPEF, respectively.

**Figure 8:** Spatially resolved maps of INAG for samples aged 24 (a) and 60 (b). Both maps share the same color bar. The inset indicates the mean value across the entire images with the corresponding standard deviation. The color bar is shown at the right.

**Figure 9:** Relationship between INAG values and age. Each symbol corresponds to the mean value for each specimen across all imaged dentinal areas. Error bars indicate the standard deviation. Black line represents the best linear fit to the data (INAG = −0.003^∗^age − 0.25).

**Figure 10:** Polarimetric SHG images for two dental pieces (dentinal area, aged 19 and 60). Each image was acquired with a different incident linear polarization states (see labels at the top of each image). Bar length: 50 *μ*m.

**Figure 11:** Maps of *ρ* computed from the images of Figure 9. Color code is shown at the right.

**Figure 12:** Relationship between *ρ* and age (*ρ* = –0.02,·age–1.03). Each symbol indicates the mean value for each specimen. Error bars indicate the standard deviation.

The article "Dental Age Estimation Using Multiphoton Microscopy: A Potential Tool for Forensic Science" was published in 2022. Journal: Biomed Res Int.

## Data Availability

The datasets used within this paper are available from the corresponding author upon reasonable request.
